# Dynamic cord compression induced by proximal junctional failure and loose pedicle screws after thoracolumbar fusion surgery: a case report

**DOI:** 10.1186/s12891-023-06791-2

**Published:** 2023-08-24

**Authors:** Takahiro Kozaki, Takuhei Kozaki, Keiji Nagata, Shunji Tsutsui, Yusuke Noda, Howard S An, Hiroshi Yamada

**Affiliations:** 1 Department of Orthopaedic Surgery, Wakayama Medical University, 811-1 Kimiidera, Wakayama, 641-0012 Japan; 2 Department of Orthopaedic Surgery, Rush University Medical Center, 1611 W. Harrison St, Chicago, IL 60612 USA

**Keywords:** Adult spinal deformity, Proximal junctional failure, Dynamic cord compression, Pedicle screw loosening

## Abstract

**Background:**

One of the common mechanical complications following spinal fusion surgery is proximal junctional failure (PJF). The incidence of neurological deficit associated with PJF has been poorly described in the literature. Here, we report a case in which numbness in the lower extremities was recognized as the first symptom, but the discrepancy in the imaging findings made PJF difficult to diagnose.

**Methods:**

A 71-year-old female underwent corrective fusion surgery. Three weeks later, she complained of persistent right leg numbness. Standing X-ray showed the back-out of the pedicle screws (PSs) in the upper instrumented vertebra (UIV), but there was no obvious evidence of cord compression on computed tomography (CT), which caused the delay of diagnosis. Five weeks later, magnetic resonance image (MRI) did not show cord compression on an axial view, but there were signal changes in the spinal cord.

**Results:**

The first reason for the delayed diagnosis was the lack of awareness that leg numbness could occur as the first symptom of PJF. The second problem was the lack of evidence for spinal cord compression in various imaging tests. Loosened PSs were dislocated on standing, but were back to their original position on supine position. In our case, these contradictory images led to a delay in diagnosis.

**Conclusion:**

Loosened PSs caused dynamic cord compression due to repeated deviation and reduction. Supine and standing radiographs may be an important tool in the diagnosis of PJF induced by dynamic cord compression.

## Background

Adult spinal deformity (ASD) has become a common spinal disorder in the aging population. Patients with ASD often present with severe low back pain and a diminished quality of life. Accordingly, the number of surgical procedures for ASD with the aim of reducing pain and improving the quality of life has increased. However, the surgical treatment for ASD is a major undertaking that can be accompanied by a wide range of postoperative complications [1–3]. One of the most common mechanical complications following spinal fusion surgery is proximal junctional kyphosis (PJK) [1]. Some studies have reported that the occurrence of PJK ranges from 20 to 61% [4–6] and causes degenerative changes or fracture at the proximal level next to the fusion segments [7, 8]. PJK is often problematic and can adversely influence the functional and neurological outcomes, and often requires further surgical intervention [9]. Preventing mechanical complications is a key factor in maintaining good radiological and clinical outcomes [10–12].

Proximal junctional failure (PJF) is often induced by fractures of the upper instrumented vertebra (UIV) and/or posterior complex of the ligaments. In severe cases, myelopathy can occur from cord compression [13]. PJF frequently requires surgical revision for correction and decompression of the spinal cord. The rate of PJF following surgery for ASD varies widely in the literature and is estimated to be between 1% and 35% [11, 14]. The incidence of neurological deficit associated with PJF has been poorly described. One study reported a rate of myelopathy following PJF or PJK was 11.4% [14]. Delayed diagnosis is likely to cause permanent paralysis, and several preventive methods have been reported [15]. PJF with myelopathy should be diagnosed and surgically corrected early to minimize permanent neurological injury [13].

Here, we report a case in which numbness in the lower extremities was recognized as the first symptom of PJF with myelopathy, but the diagnosis was delayed because of the lack of evidence of spinal cord compression on static images.

## Case presentation

A 71-year-old woman presented with low back pain related to kyphoscoliosis and flat back syndrome. She had a past medical history of osteoporosis (bone mineral density: 0.633 g/cm^2^, T score: − 2.5) and osteoporotic vertebral fracture at L2. She underwent corrective fusion surgery involving T10 to sacrum fusion with instrumentation including iliac fixation (Fig. 1). The preoperative parameters were: lumbar lordosis, 7°; sacral slope, 30°; sagittal vertical axis, 252 mm; and thoracic kyphosis, 23°. The pelvic incidence was 75°.

**Fig. 1:** Standing X-ray before (a, b) and during (c, d) the operation

The patient started walking with the help of several assistants 5 days after surgery. Three weeks later, she complained of persistent right leg numbness. A standing X-ray showed back-out of the pedicle screws (PSs) in the UIV at T10 (Fig. 2a, b). However, there was no obvious evidence of cord compression on computed tomography (CT) (Fig. 2c). Five weeks later, the numbness had worsened and extended from the right sole and dorsum of her foot through the entire lower extremity up to her groin. In addition, she developed muscle weakness in her left lower leg. Manual muscle test results were as follows: quadriceps, 2/2 (right/left); tibialis anterior muscle, 2/3; gastrocnemius, 2/3; extensor hallucis longus, 2/2; and flexor hallucis longus, 2/2. Both sides of the patellar tendon exhibited hyperflexion. There were no urinary symptoms. Magnetic resonance imaging (MRI) showed no obvious cord compression in the axial view, but there was a hyperintense signal change in the spinal cord at the level of T10 in the T2-weighted sagittal image (Fig. 2d, e).

**Fig. 2:** Standing X-ray 1 week after surgery showing back-out of the pedicle screws at the upper instrumented vertebrae (a, b). Computed tomography showing a clear zone around the loosened pedicle screws but no migration into the spinal canal (c). Magnetic resonance imaging also showed that the pedicle screws did not compress on the spinal cord in the axial view (d). However, several signal changes in the spinal cord were visible in the sagittal view (e)

We suspected the pathology involved dynamic cord compression induced by loosening of the PSs. The patient underwent revision surgery to remove the loosened PSs at T10 and to extend the fusion and fixation to T5 (Fig. 3). The patient was placed carefully in the prone position during surgery, and we checked to ensure there were no differences in the transcranial motor evoked potentials between the supine and prone positions. Following this procedure, her leg weakness and numbness improved. She had no neurological symptoms 1 year after surgery.

**Fig. 3:** Standing X-ray after revision surgery. We removed the loosened pedicle screws at T10 and extended the fusion surgery to T5

## Discussion

We have described a rare case of spinal cord compression induced by loosening of the PSs in the UIV following ASD surgery. The standing images showed back-out of the loosened PSs, but no compression of the spinal cord was visible on supine MRI and CT. This lack of compression contributed to the delay in the diagnosis and revision surgery despite progression of the patient’s neurological symptoms. This case illustrates the importance of recognizing the dynamic aspect of PJF, which can lead to neurological impairment if left untreated.

The first reason for the delayed diagnosis was the lack of awareness that unilateral foot numbness can occur as the first symptom of thoracic myelopathy associated with PJF. There is no report in the literature of foot numbness as the initial presenting symptom caused by spinal cord compression following PJK. Preoperative predictors of PJK and PJF have been studied extensively. The risk factors for PJK and PJF include advanced age, low bone quality, postmenopausal status, preoperative sagittal imbalance, severity of thoracic kyphosis, and preoperative pelvic incidence and lumbar lordosis mismatch [16–18]. Our patient displayed these risk factors.

Previous reports have shown that the presenting symptoms of PJK and PJF are mostly back pain, metal prominence at the UIV, and recurrent kyphotic deformity caused by loosening and back-out of the proximal screws and implants [19, 20]. Neurological deficits associated with spinal cord compression at the lower thoracic segments include muscle weakness and numbness of the lower extremities and possible bowel and bladder dysfunction. However, this patient initially presented with only unilateral foot numbness.

Previous studies have reported that the spinothalamic tract on the lateral side of the spinal cord can cause symptoms in the lower limbs [21]. The sacral segments are located at the most lateral component of the spinothalamic tract, and the lumbar and thoracic components are arranged in that order and proceed medially toward the central canal of the thoracic spine [22, 23]. Similarly, the corticospinal tract comprises the cervical, thoracic, lumbar, and sacral segments from the inside at the thoracic lesion [22, 23]. Therefore, in this case, the loosened PSs may have caused impingement in the lumbar and sacral regions of the lateral side of the spinal cord or the distal lumbar and sacral tracts within the spinal cord. The loosening of the PSs may have shifted them from the pedicle into the spinal canal and compressed the lateral side of the spinal cord.

The second problem was the lack of evidence for spinal cord compression on various imaging tests. The diagnosis of spinal cord compression associated with PJF is relatively straightforward on MRI. One of the causes of PJF is adjacent vertebral body fracture and intervertebral disc herniation. The intervertebral disc above the UIV withstands excess stress and, as a result, the intervertebral disc may rupture or the vertebral body may fracture, and the ligamentum flavum may buckle from the dorsal side, which compresses the spinal cord.

MRI and CT are accurate for assessing changes in the intervertebral disc, fracture, and associated spinal cord compression and cord edema [19, 24]. However, one study reported that supine MRI and CT may miss the spinal cord compression induced by dynamic instability [25]. The authors of that study reported two cases in which long thoracic fusion surgery induced a vertebral fracture at the distal side that was accompanied by dynamic instability. Supine imaging showed almost normal alignment, but a sitting X-ray revealed severe kyphotic alignment [25]. Another study reported that long thoracolumbar fusion surgery in a patient with diffuse idiopathic skeletal hyperostosis caused PJF or fracture and more severe dynamic instability [26]. The extension radiograph in that study showed normal alignment, but an X-ray in the flexed position showed subluxation and severe kyphotic posture. In our case, a standing X-ray showed back-out of the loosening PSs, but the CT and MRI, which were both taken in the supine position, showed no evidence of screw penetration into the canal or cord compression. It is likely that the loosened PSs were displaced into the canal and caused repeated spinal cord impingement or contusion during standing and trunk movement in this patient.

## Conclusions

We have described a case of PJF following surgery for ASD in which numbness in the lower extremity was initially the only symptom recognized. The diagnosis of spinal cord compression was delayed because of the apparent lack of spinal canal stenosis or screw impingement on static images. This pathology was thought to result from the loosened PSs at the UIV, which caused dynamic cord compression. In this case, the reoperation fortunately helped to restore spinal cord function; however, a missed or delayed diagnosis might result in permanent spinal cord dysfunction in other patients. This case report illustrates the importance of assessing the patient’s postoperative complaints, such as numbness in the extremity, which may result from thoracic spinal cord compression. If the neurological symptom persists, the clinician should consider spinal cord compression associated with PJF in patients who have received long fusion constructs. Seemingly normal MRI or CT results do not necessarily rule out spinal cord compression caused by dynamic instability. Whenever possible, supine and standing radiographs should be obtained along with static MRI/CT to allow the prompt diagnosis of spinal cord compression.

## Data Availability

The datasets used and/or analysed during the current study available from the corresponding author on reasonable request.
